# An Approach to Intelligent Fault Diagnosis of Cryocooler Using Time-Frequency Image and CNN

**DOI:** 10.1155/2022/1754726

**Published:** 2022-05-02

**Authors:** Sheng Gao, Zhenhua Jiang, Shaoshuai Liu

**Affiliations:** ^1^Shanghai Institute of Technical Physics, Chinese Academy of Sciences, Shanghai 200083, China; ^2^University of the Chinese Academy of Sciences, Beijing 100049, China

## Abstract

Cryocooler plays an essential role in the field of infrared remote sensing. Linear compressor, as the power component of the cryocooler, will directly affect the normal operation and performance of the detector if there is a fault. Therefore, the intelligent fault diagnosis of the linear compressor is of great significance. An intelligent fault diagnosis method based on time-frequency image and convolutional neural network is proposed to solve the problems of piston and cylinder friction, mass imbalance, and plate spring distortion in the linear compressor. Firstly, the wavelet transform time-frequency analysis method is used to generate the corresponding time-frequency image. Convolutional neural network (CNN) is used to automatically extract features of time-frequency images, so as to realize the classification of various fault modes. The results of simulation experiments show that the method can identify several fault modes of the linear compressor with 95% accuracy.

## 1. Introduction

With linear motor drive, plate spring support and gap seal technology are used to ensure long life and high reliable application requirements for the compressor [1–3]. As the main moving parts of the linear compressor, piston, plate spring, and coil are considered the core of the linear compressor which are most vulnerable to failure. It is very important to identify and locate the faults of the linear compressor accurately and quickly to prevent the failure of the linear compressor [4–6].

At present, the fault diagnosis of mechanical equipment is mainly focused on rotary machinery, and reciprocating compressor mechanical fault diagnosis work is relatively few. Vibration analysis is widely used in the field of mechanical equipment fault diagnosis. The traditional fault diagnosis methods mainly use signal processing methods such as fast Fourier transform (FFT) and short-time Fourier transform (STFT) to extract fault features. Intelligent fault diagnosis is a new developing direction of mechanical fault diagnosis. Artificial neural network and support vector machine are the two most popular methods. For example, Jamadar et al. extracted 24-dimensional characteristic parameters to describe the working state of the bearing and adopted BP neural network to classify various faults. Ali used two new features and 17 characteristic parameters to judge the health state of the bearing and then established an artificial neural network (ANN) to identify fault types. Chen et al. proposed a feature extraction and selection method and applied ANN to the diagnosis of fault severity. But the construction of eigenvectors is affected by the uncertainty and bias of domain experts.

In this context, deep learning comes into play, and its main benefit is that the deep learning approach is able to learn the nonlinear representation of the raw signal to a higher level of abstraction and complexity that is independent of the contact with the human engineer guiding the learning. Since 2015, deep learning has been successfully applied to the diagnosis or classification of vibration signals of mechanical equipment [7]. Wang et al. proposed to use wavelet scale image as the input of CNN and used a series of 32 × 32 images to detect faults in a group of vibration data. Li et al. studied the effect of a raw signal containing noise effect on CNN training. The time-frequency image obtained by the short-time Fourier transform is used as the input layer of the CNN. For the gearbox vibration data, Chen et al. input the traditional feature structure as the feature vector into the convolutional neural network (CNN) structure composed of a convolutional layer and a pooling layer.

A diagnosis method based on time-frequency image and convolutional neural network is proposed for linear compressor faults. The main structure consists of two-layer convolution layer and two-layer pooling layer. Continuous wavelet transform is used as image input of convolutional neural network. This method is selected because it provides suitable output for complex high-dimensional representation without additional feature extraction [8–10].

The rest of this article is organized as follows.  Section 1 provides an overview of deep learning and CNN.  Section 2 gives a brief overview of the basic principles of the time-frequency analysis method of continuous wavelet transform.  Section 3 outlines the CNN architecture built to complete the diagnostic task of fault detection.  Section 4 summarizes the results of applying this method to the measured linear compressor fault dataset.

## 2. Convolutional Neural Network

In the CNN structure, a neuron area in the input layer is connected to a neuron in the hidden layer, which is called the local receptive field. For each neuron in the hidden layer, the local receptive field and bias are the same. Different from traditional neural networks, CNN shares weights and deviations in the whole input layer and hidden layer. The mathematical expression of weight sharing filtering is shown in the following formula:

(1) $$\begin{array}{c} y_{ij}=\sigma \left(b+\sum_{l=0}^{n-1}\sum_{l=0}^{n-1}W_{l,m}a_{j+l,k+m}\right), \end{array}$$

where *W*_*l*,*m*_ represents the shared weight, *b* represents the deviation, *a*_*j*+*l*,*k*+*m*_ is the input activation value at a certain position, and *n* is the size of the filter.

Pooling layer is usually followed by a pooling layer in each convolutional layer, which can increase the robustness of the network while reducing the input size and network parameters of the next layer. The network structure proposed in this paper uses maximum pooling to extract features. For the convolution layer, if there are *M* feature mappings as input and *N* filters, then the output mapping of the *x*_*j*_^*l*^ layer can be calculated according to the following formula:

(2) $$\begin{array}{c} x_{j}^{l}=f\left(\sum_{i=1}^{M}x_{i}^{l-1}*k_{ij}^{l}+b_{j}^{l}\right),\;j=1,\ldots ,N, \end{array}$$

where *f* represents the activation function; *x*_*i*_^*l*−1^ is the *i*-th feature map; *k*_*ij*_^*l*^ is the *j*-th filter kernel connected to the *i*-th input mapping; and *b*_*j*_^*l*^ represents the bias corresponding to the *j*-th filter. Thus, *N* feature maps are obtained as the output. Assuming the filter size is *s* × *s*, we can use formula (3) to calculate the number of all parameters of the convolution layer:

(3) $$\begin{array}{c} P=N\times \left(s\times s\times M+1\right). \end{array}$$

The convolution operation is shown in Figure 1. After the convolution operation and adding the corresponding bias, an activation function is used to calculate the output mapping. The commonly used activation functions of neural network include logistic function, hyperbolic tangent function, and rectifying linear unit (ReLU) function, as shown in equations (4)–(6):

(4) $$\begin{array}{c} f\left(x\right)={\left(1+e^{-x}\right)}^{-1}, \end{array}$$

(5) $$\begin{array}{c} f\left(x\right)=\tanh\left(x\right), \end{array}$$

(6) $$\begin{array}{c} f\left(x\right)=\max\left(0,x\right). \end{array}$$

There are two types of pooling operations: maximum pooling and average pooling. The maximum value of the local region in the feature map is calculated by maximum pooling, and the average pooling unit is calculated by average of this region. The operation process of pooling is shown in Figure 2.

After the input image is extracted by multilayer convolutional layer and pooling layer, the obtained feature map is input to the full-connection layer for further feature extraction. In the whole convolutional neural network structure, softmax is used as a “classifier” to realize the classification of fault signals.

## 3. Time-Frequency Analysis Method

The time-frequency transform represents the joint distribution information of the signal in time and frequency at the same time. Because the fault vibration signal of linear compressor is nonstationary, the traditional frequency analysis method is unable to obtain fault characteristic information comprehensively. The time-frequency analysis method has good effect on nonstationary signal processing. The commonly used time-frequency analysis methods are wavelet transform, short-time Fourier transform, s-transform, and so on [11–14].

### 3.1. Wavelet Transformation

The CWT of signal *x*(*t*) can be realized by the convolution operation of signal *x*(*t*) and complex conjugate of a set of wavelets, whose expression is as follows:

(7) $$\begin{array}{c} W\left(\alpha ,b\right)=\frac{1}{\sqrt{\alpha }}\int s\left(t\right)\psi^{*}\left(\frac{t-b}{\alpha }\right)\text{d}t, \end{array}$$

where *α* and *b* represent expansion and translation factors, respectively. *ψ*^*∗*^(•) is the complex conjugate of the scaling and translation wavelet functions *ψ*(•). According to the definition of wavelet transform:

(8) $$\begin{array}{c} \langle x\left(t\right),x\left(t\right)\rangle =\int_{-\infty }^{\infty }{\left|x\left(t\right)\right|}^{2}\text{d}t=\frac{1}{C_{\psi }}\int_{-\infty }^{\infty }s^{-2}{\int_{-\infty }^{\infty }\left|wt\left(s,\tau \right)\right|}^{2}\text{d}s\text{d}\tau , \end{array}$$

where *C*_*ψ*_ is a constant; |*wt*(*s*, *τ*)|^2^/*C*_*ψ*_*s*^2^ can be regarded as the energy density function of the time-scale plane; and |*wt*(*s*, *τ*)|^2^Δ*s*Δ*τ*/*C*_*ψ*_*s*^2^ represents the total energy in the domain centered at time intervals Δ*s* and scale intervals Δ*τ*, which is centered on point (*s*, *τ*).

The difference between CWT and Fourier transform is that in CWT, the wavelet family replaces the sines and cosines in the Fourier transform as the basis function. Because the family of wavelets contains two parameters (expansion factor and translation factor b), a signal with a family of wavelets can be projected onto a two-dimensional, time-scale plane rather than converted into a one-dimensional plane using the Fourier transform. The wavelet coefficient *W*(*α*, *b*) represents the signal *s*(*t*) and the similarity measurement of the analysis wavelet *ψ*(*t*) at a series of different scales defined by the parameter *α* and at different time positions defined by the parameter *b*. The above formula indicates that wavelet analysis belongs to time-frequency analysis, or more appropriately, time-scale analysis, which can reflect time-frequency information of signals. Therefore, it is widely used in the field of unsteady signal analysis and mechanical equipment fault diagnosis.

### 3.2. Time-Frequency Analysis of Linear Compressor Based on Continuous Wavelet Transform

The input of the convolutional neural network structure proposed in this paper is a two-dimensional grayscale graph. Therefore, it is necessary to first convert the original vibration signal into time-frequency diagram for the six common linear compressors: normal state, mass imbalance of the rotor (slight), mass imbalance of the rotor (moderate), mass imbalance of the rotor (severe), dynamic and static friction, and plate spring distortion. The time-frequency graphs corresponding to them are converted by continuous wavelet transform, as shown in Figure 3.

## 4. Data Preprocessing and the Proposed CNN Structure for Linear Compressor Fault Diagnosis

### 4.1. Data Preprocessing

The method proposed in this paper needs to preprocess the original data and convert them into image format. The input of CNN should be in the form of *m* × *n* × *k* matrix. In the field of image processing, the value of *k* is usually 3, representing the three channels of the color image. In order to simplify the calculation, this paper adopts the grayscale graph as the input, so the value of *k* is 1. This paper uses the time-frequency analysis method of wavelet transform, and the specific operation is shown in Figure 4.

Firstly, the original signal is converted into time-frequency graph by wavelet transform. The information content of color pictures is too large, and when the picture is recognized, it is actually enough to use the information in the grayscale image, so the purpose of image grayscale is to improve the speed of operation. Then, MATLAB was used to convert the time-frequency diagram into a grayscale diagram. To reduce the computational load and facilitate CNN training, the image size was compressed to 32 × 32.

### 4.2. Proposed CNN Structure

Based on the limited amount of data and insufficient computing power, the network we designed is not complicated. As shown in Figure 5, C1 is the first convolutional layer. The number of convolution kernels is 6, and the size of convolution kernels is 5 × 5; P1 represents the pooling layer of the first layer. The pooling layer adopts the maximum pooling method, and the size of the pooling area is 2 × 2. C2 represents the second convolution layer, the number of convolution kernel is 12, and the size of convolution kernel is 5 × 5; P2 represents the second pooling layer, which adopts the maximum pooling, and the size of the pooling area is 2 × 2. *F* is a fully connected layer with 120 nodes, and softmax is the output layer that contains six classes. Softmax sorter was used and drop technology was used in the whole connection layer (*p* was set to 0.4). The training model adopts the small batch gradient descent method with batch size of 50 and learning rate of 0.01, so as to minimize the cross entropy loss.

## 5. Experiment Research

### 5.1. Fault Data Acquisition and Analysis

In order to verify the superiority and effectiveness of the proposed method, the experimental data in this paper were collected from the simulation test platform for fault diagnosis of small cryogenic refrigerator designed by Shanghai Institute of Technology, Chinese Academy of Sciences, as shown in Figure 6. The fault test used acceleration sensor and data acquisition software of mpichina company in Germany. The sampling frequency is 1024 Hz, and the sampling time is 2 s, that is, 2048 points are sampled at one time. The vibration data of the refrigerator under six fault states were tested: normal state, mass imbalance of the rotor (slight), mass imbalance of the rotor (moderate), mass imbalance of the rotor (severe), dynamic and static friction, and plate spring distortion, as shown in Table 1. In each test, a single failure is guaranteed while other parts are normal.

Mass imbalance fault of the rotor is due to machining errors and prolonged wear. For the mass imbalance fault of the rotor, 20 g, 40 g, and 60 g mass blocks are added on the piston connecting rod at one end of the linear compressor to realize the mass imbalance of the motors on both sides of the linear compressor. The dynamic and static rubbing fault is due to the small gap between the two and the contact. The dynamic and static rubbing fault is achieved by changing the piston and the inclination angle between the piston and the cylinder. The clearance between the piston and the cylinder is usually only 10 to 20 microns. Due to the small gap between the piston cylinders, when the cylinder is skewed or there is debris, it will cause friction between the piston and the cylinder. The friction between the piston and the cylinder can be realized by controlling the piston's inclination angle. For the plate spring distortion fault, when installing the single motor plate spring, loosen the nut of the outer plate spring, tighten the center nut with torque wrench to make the plate spring twisted, and then lock the nut of the outer ring.

The fault diagnosis process of linear compressor is shown in Figure 7. 1000 samples are collected for each fault, and each signal length is 2 s. 70% data are randomly selected as training samples, and 30% data are selected as test samples.

### 5.2. Parameter Selection of CNN

The selection of appropriate parameters is very important for the training of CNN. For different sample sets, the selection of optimal parameters is also different. When training CNN, it is an important program to find the optimal parameter of corresponding dataset.

#### 5.2.1. Learning Rate

In the process of CNN training, stochastic gradient descent (SGD) is selected as the optimizer, and the learning rate is a very important parameter, which directly affects the updation of weights and error convergence [15]. Therefore, choosing an appropriate learning rate is crucial to improve the efficiency of network training. Setting a large learning rate at the beginning speeds up convergence and avoids getting stuck in local minima, and then a small learning rate is set so that the model can converge. In the process of CNN training, the optimal learning rate was selected by comparing the loss and accuracy under different learning rates. The results are shown in Table 2.

According to the analysis of Table 2 and Figure 8, with the increase of learning rate, the training accuracy and test accuracy increase. When the learning rate increases to 0.001, the accuracy reaches the maximum; when the learning rate continues to increase, the accuracy decreases. Therefore, the learning rate proposed in this paper is equal to 0.001.

#### 5.2.2. Batch Size

In the training of CNN, due to the large amount of sample data, limited computer configuration, and other conditions, we cannot let all the samples be used for network training at the same time. Therefore, it is usually best to divide the sample into medium-sized chunks.

The size of this block is called the batch size. In this experiment, we used different batch sizes to train CNN, and other parameters were the same. Losses, accuracies, and time costs are shown in Table 3.

It can be known from Figures 9 and 10 that the smaller the batch size is, the higher the prediction accuracy will be and the longer the iterative calculation time will be. When the value of batch size is 10, the accuracy decreases less when comparing smaller size, and the training time decreases to a greater extent. When the value is greater than 10, the prediction accuracy decreases greatly, but the training time does not decrease significantly. To sum up, when the batch size of the CNN structural training parameter proposed in this paper is equal to 10, both the prediction accuracy and the training time are taken into account.

Input the grayscale image into the CNN structure proposed in this paper and take the learning rate equal to 0.001 and the batch size equal to 10. The final predicted results are shown in Figure 11. The abscissa is shown from left to right: normal state, mass imbalance of the rotor (slight), mass imbalance of the rotor (moderate), mass imbalance of the rotor (severe), dynamic and static friction, and spring distortion.

Using the CNN structure and the optimized parameters, the recognition rate of the six states of the linear compressor is increased to 95.5%.

## 6. Conclusion

Obviously, the following conclusions can be drawn from the above analysis results. By using WPT to transform the original vibration signal into time-frequency diagram, more and richer fault information can be obtained. At the same time, it avoids the tedious manual extraction and selection of fault features and simplifies the fault diagnosis program. Secondly, the optimized structural parameters of CNN can improve the fault identification accuracy to 95.5% and shorten the training time. The validity of the method is verified by the measured fault data of the linear compressor.

Future work will include more experimental tests to further understand the limitations of CWT and CNN methods [16–18], especially for some more complex failures, such as multiple failures occurring simultaneously and coupling with each other. For the determination of optimal parameters, it is still a problem to be further studied; especially when using a deeper network structure or studying another completely different fault, the corresponding optimal parameters may also change.

## Figures and Tables

**Figure 1:** Convolution operation.

**Figure 2:** Two pooling operations.

**Figure 3:** Time-frequency diagram of different states of compressor. (a) Normal state of the linear compressor. (b) Mass imbalance (slight). (c) Mass imbalance (moderate). (d) Mass imbalance (severe). (e) Dynamic and static friction. (f) Plate spring twist.

**Figure 4:** The time-frequency transform and grayscale.

**Figure 5:** Proposed CNN structure.

**Figure 6:** Linear compressor diagnostic simulator system.

**Figure 7:** Flowchart of linear compressor fault diagnosis.

**Figure 8:** Accuracy under different learning rates.

**Figure 9:** Accuracy under different batch sizes.

**Figure 10:** Time cost under different batch sizes.

**Figure 11:** Accuracy of the proposed CNN structure.

**Table 1:** Six linear compressor states.

Linear compressor states	Number of samples	The label	Hot coding alone
Normal state	1000	1	100000
Mass imbalance (slight)	1000	2	010000
Mass imbalance (moderate)	1000	3	001000
Mass imbalance (severe)	1000	4	000100
Dynamic and static friction	1000	5	000010
Plate spring twist	1000	6	000001

**Table 2:** Accuracy under different learning rates.

Learning rate	Train loss	Test loss	Train accuracy	Test accuracy
0.0001	1.4535	1.4129	0.5627	0.5426
0.0005	0.1935	0.1752	0.9019	0.9098
0.0008	0.1237	0.1216	0.9126	0.9218
0.0009	0.0924	0.0919	0.9244	0.9315
0.001	0.0831	0.0842	0.94	0.9498
0.0015	0.1016	0.1024	0.6802	0.6794
0.002	0.9812	0.9655	0.5924	0.5996
0.005	1.5534	0.5167	0.3202	0.3228
0.01	1.5611	0.5098	0.5112	0.3155

**Table 3:** Accuracy and time cost under different batch sizes.

Batch size	Train accuracy	Test accuracy	Time cost (s)
8	0.9488	0.9535	325
16	0.9362	0.9528	181
32	0.9532	0.9478	121
64	0.9298	0.9419	100
20	0.8521	0.8645	89
40	0.7756	0.8025	80

## Data Availability

The data used to support the findings of this study are available from the corresponding author upon request.
